The article "The effect of early oral stimulation with breast milk on the feeding behavior of infants after congenital cardiac surgery" was retracted in 2023. Reason: lack of ethics approval or compliance.

# The effect of early oral stimulation with breast milk on the feeding behavior of infants after congenital cardiac surgery

**DOI:** 10.1186/s13019-020-01355-0

**Published:** 2020-10-09

**Authors:** Xian-Rong Yu, Shu-Ting Huang, Ning Xu, Li-Wen Wang, Zeng-Chun Wang, Hua Cao, Qiang Chen

**Affiliations:** 1 Department of Cardiac Surgery, Fujian Maternity and Child Health Hospital, Affiliated Hospital of Fujian Medical University, Fuzhou, China; 2 Fujian Key Laboratory of Women and Children’s Critical Diseases Research, Fujian Maternity and Child Health Hospital, Fuzhou, China; 3 Department of Cardiovascular Surgery, Union Hospital, Fujian Medical University, Fuzhou, China

**Keywords:** Breast milk, Breast milk oral stimulation, Infant, CHD

## Abstract

**Objective:**

To investigate the effect of early oral stimulation with breast milk on the feeding behavior of infants after congenital cardiac surgery.

**Methods:**

Infants with congenital heart disease were randomly divided into the breast milk oral stimulation group (*n* = 23), physiological saline oral stimulation group (*n* = 23) and control group (*n* = 23). Debra Beckman’s oral exercise program was used with breast milk and physiological saline in the breast milk oral stimulation group and the physiological saline oral stimulation group, respectively. The time oral feeding and total oral nutrition were started, the length of intensive care unit (ICU) stay and hospital stay, weight and the complications at discharge were recorded for each group and statistically analyzed.

**Results:**

The time oral feeding and total oral nutrition were started and the length of ICU stay and hospital stay were significantly less in the breast milk oral stimulation group and physiological saline oral stimulation group than in the control group (*P* < 0.05). There were no significant differences in other indicators between the breast milk oral stimulation group and the physiological saline oral stimulation group, except for the time total oral nutrition began (*P* < 0.05). However, there were no significant differences in weight or complications at discharge among the three groups (*P* > 0.05).

**Conclusion:**

Early oral stimulation exercises with breast milk can help infant patients quickly recover total oral nutrition and reduce the length of ICU and hospital stay after cardiac surgery.

## Introduction

With improvements in prenatal diagnosis, cardiac surgery technology and perioperative intensive care, the survival rate of infant patients with congenital heart disease (CHD) has significantly improved [1]. In the perioperative period, the role of feeding in infants after cardiac surgery has become increasingly prominent, and nutrition is another main focus, aside from the maintenance of cardiopulmonary function and the prevention of postoperative complications [2]. After cardiac surgery associated with cardiopulmonary bypass, infants’ body functions may be impaired to some extent, including renal insufficiency, gastrointestinal dysfunction and swallowing dysfunction [3]. Gastrointestinal dysfunction and swallowing dysfunction prevent the early establishment of total oral nutrition, which may affect the postoperative recovery of patients. Studies have shown that early oral stimulation of infants with gastrointestinal dysfunction has a significant effect on the recovery of gastrointestinal function [4, 5]. According to the literature review, no article has focused on the use of oral stimulation with breast milk in infants after cardiac surgery. This study performed early oral stimulation with breast milk on infants after cardiac surgery and evaluated the effect of such treatment on the recovery of gastrointestinal function in those infants.

## Methods

This study was approved by the ethics committee of Fujian Medical University and our hospital, and informed consent was obtained from the families of all patients who participated in the study. According to the mean (12.5, 13.1, 16.2) and standard deviation (3.1, 3.9, 4.0) of the length of hospital stay in the presurvey, with α = 0.05, a two-tailed test and a power of 90%, the sample size of the three groups was 23; the sample size was calculated with SPSS software package version 16.0. The inclusion criteria were as follows: 1. infant patients after cardiac surgery. 2. satisfactory surgical results and stable hemodynamics. The exclusion criteria were as follows: 1. associated with other structural and functional abnormalities (such as esophageal atresia, esophageal hiatal hernia, poor bowel rotation, etc.). 2. family members of the patients declined to participate in the study.

This study was completed in the cardiac intensive care unit (ICU) of a provincial teaching hospital. The clinical data of 69 infant patients with CHD who underwent cardiac surgery with cardiopulmonary bypass in our hospital from January 2020 to June 2020 were collected. During the same period, 74 patients received cardiac surgery in our hospital, and 5 patients were excluded from the group, among which 2 patients had congenital intestinal malformations and the other 3 patients’ family members refused to participate in this study. All eligible patients were randomly divided into the breast milk oral stimulation group (*n* = 23), the physiological saline oral stimulation group (*n* = 23) and the control group (*n* = 23) based on a set of random numbers generated by a computer. All patients consulted with an otolaryngologist before surgical correction to confirm the absence of ears, nose and throat structure deformity. General clinical data of all groups are shown in Table 1.

**Table 1:** Comparison of the general data between the three groups

	Breast milk oral stimulation group	Physiological saline oral stimulation group	Control group	*P* values
Age (month)	1.4 ± 1.1	1.5 ± 1.3	1.6 ± 1.2	0.698
Weight (kg)	3.7 ± 1.3	3.6 ± 1.5	3.8 ± 1.4	0.672
Male/Female	10/13	12/11	11/12	0.840
Disease				
Ventricular septal defect	15	16	15	0.974
Pulmonary stenosis	3	2	3	
Coarctation of aorta	1	1	2	
Total anomalous pulmonary venous connection	3	2	1	
Interrupted aortic arch	1	2	2	
Preoperative complications				
Pneumonia	2	4	4	0.231
Liver insufficiency	1	0	0	–
Renal insufficiency	0	0	0	–
Operation time (h)	3.8 ± 1.2	3.7 ± 1.6	3.8 ± 1.4	0.343
Cardiopulmonary bypass time (h)	1.8 ± 0.9	1.9 ± 0.7	1.9 ± 0.8	0.547
Aortic cross-clamping time (h)	1.1 ± 0.4	1.0 ± 0.7	1.1 ± 0.3	0.754

In the breast milk oral stimulation group and the physiological saline oral stimulation group, the early oral exercise stimulation program was performed by a professional infant rehabilitation physician from our hospital using Debra Beckman’s oral exercise program with breast milk or physiological saline, respectively [6]. The specific steps were as follows: 10 min of oral stimulation with breast milk or physiological saline and physical exercise were performed on the cheeks, gums, jaws and tongue of the child; then, a nipple was used for two to 3 min of nonnutritive stimulation. The patients underwent oral stimulation with breast milk or physiological saline once a day, 6 days a week during the early postoperative period after the patients’ hemodynamics were stable, as evaluated by the cardiac surgeon. The end of oral stimulation was when the patients received total oral nutrition. No oral exercise stimulation program was performed in the control group. In the early postoperative period, oral nutrition began to be restored after the children’s hemodynamic stability and the bowel sounds returned. The principle of breastfeeding adopted in this paper was of multiple sessions of breastfeeding with a small amount of breast milk (1 ml/kg/h) to gradually restore oral nutrition for the patients in each group. If there were no symptoms such as vomiting, abdominal distension, or diarrhea, the amount of oral nutrition was gradually increased at a rate of 1 ml/kg/6 h until total oral nutrition was restored. The oral feeding regimen of the infants in each group was the same (breastfeeding).

The data of all the infant patients before and after oral treatment were evaluated and collected by the professional rehabilitation physician to ensure the reliability of the data obtained. The time oral feeding and total oral nutrition were started, the length of ICU stay and hospital stay, weight and the complications at discharge were recorded for all patients and statistically analyzed. Factors influencing the resumption of total oral nutrition and discharge were also collected.

### Statistical analysis

The continuous data are expressed as the mean ± standard deviation, and they were tested for normal distributions. An independent sample t test was used for those data with to a normal distribution, while the Wilcoxon test was used for those data without a normal distribution. Quantitative data were compared between groups by the chi-square test. *P* < 0.05 was considered statistically significant. SPSS software package version 16.0 (SPSS Inc. IBM Corporation) was used for data analysis and management.

## Results

As shown in Table 1, there were no significant differences in the general clinical data of the three groups, which indicated that the three groups of patients were homogeneous and comparable. The time oral feeding and total oral nutrition began and the length of ICU and hospital stay were significantly less in the breast milk oral stimulation group and the physiological saline oral stimulation group than in the control group (*P* < 0.05). There were no significant differences in other indicators between the breast milk oral stimulation group and the physiological saline oral stimulation group, except for the time total oral nutrition began (*P* < 0.05). There were no significant differences in weight or complications at discharge among the three groups (*P* > 0.05). (Table 2).

**Table 2:** Comparison of the postoperative date between the three groups

	Breast milk oral stimulation group	Physiological saline oral stimulation group	Control group	*P* values
The time oral feeding (h)	29.8 ± 10.2	31.7 ± 10.5	49.8 ± 11.5^*#^	0.028
Total oral nutrition time (d)	3.5 ± 0.8	4.3 ± 1.1^*^	4.9 ± 1.6^*#^	0.034
Length of intensive care unit stay (d)	4.5 ± 1.4	4.8 ± 1.7	7.8 ± 1.5^*#^	0.041
Length of hospital stay (d)	12.9 ± 3.4	13.4 ± 4.4	16.7 ± 5.2^*#^	0.043
Postoperative complications				
Pneumonia	3	3	4	0.889
Liver insufficiency	2	1	1	0.767
Necrotizing enterocolitis	0	0	0	–
Gastrointestinal hemorrhage	0	0	0	–
Death	0	0	0	–
Patients with nasogastric tube at discharge	1	1	3	0.422
Weight at discharge	4.5 ± 1.1	4.3 ± 1.3	4.4 ± 1.5	0.548

* indicates *p* < 0.05 compared with breast milk oral stimulation group,

^#^ indicates *p* < 0.05 compared with saline oral stimulation group

## Discussion

There are more postoperative complications associated with pediatric cardiac surgery than with conventional pediatric general surgery. In addition to cardiac function-related complications, systemic complications, such as abnormal liver and kidney function and impaired gastrointestinal function, often occur in the postoperative recovery stage [7, 8]. The main reason is due to the impact of cardiopulmonary bypass and intraoperative hypothermia on various organ functions. For the recovery of nutritional support after cardiac surgery in infants, in addition to overcoming the potential injury from cardiopulmonary bypass during the operation and subjection of the gastrointestinal tract to ischemia-reperfusion injury, oropharyngeal injury and swallowing dysfunction caused by tracheal intubation must also be evaluated and treated [9, 10]. If feeding disorder after cardiac surgery is avoided, patients can effectively avoid hospital complications caused by the use of total parenteral nutrition, nasogastric tubes, or even fistulas, which can even speed up the patients’ recovery process [11, 12]. Therefore, feeding and nutrition problems are particularly important of the postoperative management of infants with CHD.

Many infants with CHD require prolonged endotracheal intubation and mechanically assisted ventilation after cardiac surgery, and some of them have varying degrees of difficulty with feeding. According to a literature search, many researchers have adopted various strategies to improve oral motor function in postoperative children with feeding disorders [13, 14]. Some researchers applied nonnutritive pacifier sucking strategies when the children were in a fasting period to accelerate the maturation of sucking reflexes. This treatment promoted a rapid shift from a nonoral diet to an oral diet, possibly because it allowed the infant to engage the neuromuscular structures needed to suck with greater efficiency and endurance [15, 16]. Other scholars have demonstrated that applying mild pressure stimulation to oral muscles could significantly increase the speed of sucking per minute and the amount of milk consumed, which might be due to the stimulation strengthening the oral musculature required for adequate and efficient sucking and enhancing the maturation of central and peripheral nervous system structures, thus leading to improved sucking skills, rates of milk transfer, milk intake, and coordination of the suck-swallow-breathe reflex [17–19]. Sandra and his teams believed that oral motor stimulation could improve the performance of children after nutritional sucking, while sensory-motor-oral stimulation associated with nonnutritive sucking might increase the maturity of the neural structure, thereby improving coordination [20]. Debra Beckman’s oral exercise program combines oral stimulation and nonnutritive nipple sucking strategies and is widely used in the clinic. During feeding, perioral stimulation with rhythmic pressure is applied to the baby’s tongue, and this supports the stability of the jaw and tongue. Nonnutritive nipple sucking promotes coordination of oral movements in infants. After such treatment, infants’ oral movements significantly improve. To our knowledge, there have been no reports of early postoperative oral stimulation in infants with CHD. We adopted an oral stimulation with breast milk intervention to explore whether such an intervention was beneficial to the postoperative oral movement and gastrointestinal function recovery of these infants.

In this study, patients in the breast milk oral stimulation group and the physiological saline oral stimulation group began to perform oral stimulation with breast milk or physiological saline, respectively, during the early postoperative period when the patient’s hemodynamics were stable. The results showed that the time oral feeding and total oral nutrition started and the length of ICU stay and hospital stay were shorter in the two treatment groups than in the control group. Studies have shown that oral stimulation exercise procedures, including the promotion of nonnutritive sucking, significantly shorten the length of hospital stay of preterm infants by improving oral exercise coordination and nonnutritive sucking, which is also consistent with the results of this study [21]. Providing oral stimulation exercise with breast milk before oral nutrition has significant benefits for infants with congenital cardiac surgery in the following aspects: restoration of feeding methods, improvement of the coordination of sucking movements, increase in the amount of milk sucked, enhancement of the transition to total oral nutrition, and shortened length of hospital stay. Compared with that of the physiological saline oral stimulation group, the total oral nutrition time in the breast milk oral stimulation group was significantly reduced. The reason might be that breast milk was the most natural and safe food during the growth of infants, and it was rich in probiotics and nutrients. Using breast milk for oral stimulation could prevent imbalance of the digestive tract flora, thereby inhibiting bacterial proliferation and promoting the recovery of oral nutrition in children [22]. However, it is worth noting that there was no significant difference in weight at discharge between the three groups. It could be inferred that the recovery time of total oral nutrition in the breast milk oral stimulation group and the physiological saline oral stimulation group was shorter, and the nutritional intake was greater than that of the control group. This situation might be due to the longer length of hospital stay in the control group and the longer time for weight gain.

Only 1 infant in the breast milk oral stimulation group and 1 infant in the physiological saline oral stimulation group were still on a nasogastric tube feeding diet when they were discharged from the hospital, while there were 3 patients who remained on a nasogastric tube feeding diet at discharge in the control group. Although there was no significant difference among the three groups, this could be explained by the need for indwelling nasogastric tubes in those patients with oral stimulation training being reduced. The nasogastric tube was successfully removed in these patients after a period of outpatient follow-up treatment. Due to increased caloric requirements and delayed oral motor skills associated with long-term tracheal intubation, infant patients might need to receive nasogastric tube feeding for a long time or require other nutritional methods, which might cause oral motor development delay, increase gastroesophageal reflux, etc. [23] Studies have shown that in infants who do not have difficulty swallowing, those who have undergone early postoperative oral stimulation recovery training had indwelling gastric tubes for 3 days less than those who have not received such training [24]. These conclusions are consistent with our findings, suggesting that our interventions were effective in postoperative recovery in infant patients with CHD.

This study has some limitations. This is a single-center study with a small sample size, which may have caused case selection bias. Other centers, different populations, and different treatment plans may lead to different conclusions. Second, the research object was mainly infant patients with simple CHD and cannot represent other patients with other types of CHD, such as children with complicated CHDs. However, a larger sample size might lead to different stratification outcomes for different diseases, which could influence the conclusions. However, we believe that our conclusion still has some significance, and future research also needs to further discuss this part of the problem.

## Conclusion

Through early oral stimulation exercise with breast milk, infant patients experienced a faster recovery of gastrointestinal function and a shorter length of ICU and hospital stay after cardiac surgery. Therefore, the strategy of early oral stimulation with breast milk in the postoperative period for infant patients with congenital heart disease is worth promoting.

## Data Availability

Data sharing not applicable to this article as no data sets were generated or analyzed during the current study.

## Abbreviations

CHD: Congenital heart disease
ICU: Intensive care unit
